The article "The World Health Organization's Frontline Support to Countries During the COVID-19 Pandemic in 2020" was published in 2022. Journal: Front Public Health.

# The World Health Organization's Frontline Support to Countries During the COVID-19 Pandemic in 2020

**DOI:** 10.3389/fpubh.2022.850260

**Published:** 2022-03-18

**Authors:** Amy Coates, Kathleen Taylor Warren, Corey Henderson, Michelle McPherson, Offeibea Obubah, Peter Graaff, Shambhu Acharya

**Affiliations:** ^1^Country Strategy and Support, World Health Organization, Geneva, Switzerland; ^2^COVID-19 Country Technical Support, Health Emergencies Programme, World Health Organization, Geneva, Switzerland; ^3^Consultant, World Health Organization, Geneva, Switzerland; ^4^Health Emergencies Programme, World Health Organization, Geneva, Switzerland

**Keywords:** COVID-19, SARS-CoV-2, pandemic response, World Health Organization, World Health Organization country offices, technical assistance

## Abstract

The World Health Organization (WHO) declared the SARS-CoV-2 outbreak a Public Health Emergency of International Concern (PHEIC) on January 30, 2020. WHO rapidly scaled up its response including through its 149 country offices to support Member States prepare for and respond to the COVID-19 pandemic. This article describes the frontline role of the WHO Country Offices (WCOs) and demonstrates that WHO utilized its existing country presence to deliver its global program of work during this unprecedented emergency. Using data collected from the 2020 WHO COVID-19 Strategic Preparedness and Response Plan monitoring and evaluation framework assessments, plus data collected in a quantitative survey completed by 149 WCOs during 2020, this article describes how WHO supported national authorities and partners through leadership, policy dialogue, strategic support, technical assistance, and service delivery, in line with WHO's current 5-year strategic plan, the WHO 13th General Programme of Work 2019–2023. Country level case studies were used to further illustrate actions taken by WCOs. WHO's achievements notwithstanding, the Organization faced several key challenges in the first year of the response. Recommendations to enhance WHO presence in countries for future emergency prevention, preparedness and response, from several independent reviews, were presented to the World Health Assembly in May 2021 and relevant recommendations are presented in this article.

## Introduction

The COVID-19 pandemic has disrupted lives and livelihoods of people and communities globally, causing in excess of a reported 1.8 million deaths in 2020 (1) and contributing to millions more (1–4). After the World Health Organization (WHO) declared the SARS-CoV-2 outbreak a Public Health Emergency of International Concern (PHEIC) on January 30, 2020, WHO mobilized its global resources at an unprecedented scale, leveraging existing preparedness and response mechanisms to support country-level actions (5). WHO activated its global Incident Management System (6) to rapidly scale up its response capacities and mobilized every facet of WHO expertise to support Member States prepare for and respond to the COVID-19 pandemic (5).

The article "The World Health Organization's Frontline Support to Countries During the COVID-19 Pandemic in 2020" was published in 2022. Journal: Front Public Health.

WHO is the specialized agency of the United Nations (UN) that provides global leadership, convening and coordination on public health. WHO's role in monitoring and reporting on health security threats, setting norms and standards, issuing technical guidance and driving the research and development agenda in collaboration with the global science community in times of emergency is well-documented (7). The WHO current 5-year strategic plan, the 13th General Programme of Work 2019–2023 (GPW13) details how WHO works in and with countries (8), with the engagement between WHO and each country tailored to the specific needs, context, capacities and vulnerabilities of that country. In some settings, this engagement is upstream policy and strategy related, whereas in other countries the engagement is downstream with a focus on technical assistance and strengthening service delivery.

Despite now having a country presence in 152 countries, territories and areas (9), the role of WHO, in collaboration with partners, to support national governments to respond to the pandemic is not well documented in the published literature. This article presents the frontline role of the 149 WHO country offices (WCOs), during the first year of the COVID-19 pandemic response using three key themes aligned with the GPW13: (a) leadership, (b) policy dialogue and strategic support, and (c) technical assistance and service delivery. The WHO COVID-19 Strategic Preparedness and Response Plan (SPRP) monitoring and evaluation framework (2020) assessments, and data collected in a quantitative survey completed by 149 WCOs during the third quarter of 2020 (10) are used to describe WHO's roles and contributions in countries (summarized in Table 1). For each theme, a relevant country example was selected from published country level case studies (11–13). Most of the survey and case study data collected from WCOs was self-reported, so to maximize the quality and accuracy of reporting, and improve consistency of responses to the survey questions and interviews, two rounds of cross checking with respondents were conducted. Additional validation of survey responses and case study reports was carried out by focal points from the Country Office Support Unit Network in the six WHO Regional Offices. Challenges and recommendations for strengthening the role of WHO in health emergencies from several independent reviews (14–16) that were presented to the World Health Assembly in May 2021 are included, which are currently under consideration by a Working Group of WHO Member States (17).

The article "The World Health Organization's Frontline Support to Countries During the COVID-19 Pandemic in 2020" was published in 2022. Journal: Front Public Health.

**Table 1:** Timeline of key WHO frontline support during the first year of the COVID-19 pandemic.

**Strategic shift**	**Achievements**	**% Of countries**
**Before COVID-19 declared a PHEIC (January 30, 2020)**		
Leadership	Incident Management system activation by WCOs	22%
**Before the first case was reported in the country**		
Leadership	Incident Management system activation by WCOs	65%
Policy dialogue and strategic support	WCOs initiated support to national governments to develop a response monitoring framework	71%
Technical assistance and service delivery	WCOs provided technical assistance to national governments and partners on priority interventions related to risk communication, community engagement and disease control measures	84%
**By February 2020**		
Leadership	WCOs Initiated or supported Ministries of Health to initiate health sector cluster meetings	55%
	WCOs developed or updated business continuity plans to ensure WHO continuity of national support	100%
Policy dialogue and strategic support	WCOs had initiated support for developing CPRPs	81%
Technical assistance and service delivery	WCOs had initiated support for procurement and logistics due to the unprecedented challenges to the global supply chain caused by the COVID-19 pandemic	83%
**By the time the pandemic was characterized (March 11, 2020)**		
Leadership	Incident Management system activation by WCOs	77%
**By March 2020**		
Leadership	Countries (all member states) with an established COVID-19 response coordination mechanism	45%
Policy dialogue and strategic support	Countries (all member states) with CPRPs	46%
	WCOs had provided support to develop and disseminate regular country situation reports and bulletins to partners and the public	77%
Technical assistance and service delivery	Countries had access to laboratory testing (either in country or through an arrangement with a neighboring country)	85%
**By June 2020**		
Leadership	Countries (all member states) with an established COVID-19 response coordination mechanism	92%
Policy dialogue and strategic support	Countries (all member states) with CPRPs	83%
**By August 31, 2020**		
Leadership	WCOs coordination role within the UN country teams increased during the COVID-19 response	90%
	WCOs led the health response amongst UN partners	87%
	WCOs led the “health first” pillar of the UNs' framework for the immediate socio-economic support to countries and societies in the face of COVID-19	65%
	WCOs raised funds from donors	73%
	WCOs led national donor coordination mechanisms for the response	59%
Technical assistance and service delivery	Existing international staff in repurposed for the COVID-19 response	60%
	Countries that received in-person or virtual technical assistance from WHO experts based in regional or sub-regional offices	93%
	Countries that received in-person or virtual technical assistance from WHO experts based in WHO headquarters	74%
**By the end of 2020**		
Leadership	Countries (all member states) with an established COVID-19 response coordination mechanism	97%
	WCO implemented the majority of WHO's total funds raised globally for the COVID-19 response	67% (US$ 849.4 M)
Policy dialogue and strategic support	Countries (all member states) with CPRPs	91%
	WCO conducted intra-action reviews (IARs) of national and subnational COVID-19 responses following new guidance published July 2020.	24%
Technical assistance and service delivery	Countries able to test for SARS-CoV-2	100%
	Global Outbreak and Response Network (GOARN) and Emergency Medical Teams (EMT) mobilized for 191 deployments to countries (all member states) to provide immediate assistance, training, and support	
	Countries (all member states) where WHO procured and supplied critical COVID-19 health commodities including diagnostic tests, medical equipment and personal protective equipment	86%
**By April 2021**		
Policy dialogue and strategic support	Countries developed a package of essential health services to be maintained during the pandemic	87%
	Countries had designated a focal point for the maintenance of essential health services	82%
	Countries had allocated additional funding for the maintenance of essential health services	62%

*Denominator for all % calculations is 149 WCOs, except where stated otherwise*.

The article "The World Health Organization's Frontline Support to Countries During the COVID-19 Pandemic in 2020" was published in 2022. Journal: Front Public Health.

## Leadership

A core function of WHO is to provide leadership on matters critical to the health of all people and to convene and coordinate effective joint action of the many in-country partners (8). During the first year of the pandemic, WHO's existing country-level presence, infrastructure and established systems through the 149 WCOs enabled leadership and coordination efforts to be intensified to support country pandemic preparedness and COVID-19 response efforts.

The WHO Incident Management System was activated by 22% of WCOs before WHO declared COVID-19 a public health event of international concern (PHEIC) on January 30, 2020 and by 65% of WCOs before the first COVID-19 case was reported in the country (Table 1). When COVID-19 was characterized as a pandemic on March 11, 2020, 77% of WCOs had already activated their Incident Management System (10) (Table 1). Within weeks of the PHEIC declaration, all WCOs had business continuity plans to “ensure WHO was able to deliver swift and effective emergency response” actions in support of national plans (18).

The article "The World Health Organization's Frontline Support to Countries During the COVID-19 Pandemic in 2020" was published in 2022. Journal: Front Public Health.

To support country coordination and national response implementation, WHO built on well-established relationships with national governments and partners to support countries to activate or establish functional emergency coordination mechanisms at the national level (19). By February 2020, more than half (55%) of WCOs had initiated or supported the Ministry of Health to initiate health sector or health cluster meetings (10) (Table 1). By March 2020, 45% of countries had established a COVID-19 response coordination mechanism, which increased to 92% of countries by end June 2020 (5) and 97% of countries by the end of 2020 (Table 1). These multisectoral emergency coordination mechanisms included plans and procedures, physical infrastructure, information systems and standards, and human resources. In addition, WHO played an important leadership role within the UN System at the country-level. Most WCOs (90%) reported that their coordination role within the United Nations Country Teams increased during the COVID-19 response, with 87% also reporting they led the health response among UN partners, and 65% reporting that they led the “health first” pillar of the UNs' Framework for the Immediate Socio-Economic Support to Countries and Societies in the Face of COVID-19 (10) (Table 1).

Using its existing decentralized administration processes, WHO directed financial resources to the country level, as close to the emergency and the affected population as possible. In 2020, of the US$ 1,267.8 million funds raised and utilized for the COVID-19 response by WHO globally, 67% (849.4 million USD) was implemented by WCOs (20). Contributing to the availability of resources at country level, 73% of WCOs raised funds from donors and 59% of offices led national donor coordination mechanisms for the response (10) (Table 1).

WHO's country level leadership is illustrated in Kazakhstan (13, 21) where WHO led the UN COVID-19 response. This included establishing an inter-agency risk communication group to regularly review key messages, promote public health and social measures, and oversee and support new and innovative inter-agency logistics coordination platform to avoid duplication. The WCO raised ~US$6.2 million for the response (21) and boosted its human resources capacity from five to 22 staff for the critical support to the national response (13) in areas such as leadership and coordination, infection prevention and control, case management, laboratories, and risk communication (7).

## Policy Dialogue and Strategic Support

Policy dialogue is the communication between stakeholders to contribute to a process which culminates in a policy decision (22, 23). WCOs tailor policy dialogue to local needs and contexts to support access of national authorities and other partners and stakeholders to the latest scientific evidence, to promote and enable evidence-based decision making and implementation of WHO's normative work at the country level (8). WHO published its initial SPRP in February 2020 (24) with a revision in April 2020 (25). The SPRP and subsequent operational guidelines (26) set out the essential pillars required at the national level to “reduce transmission of the SARS-CoV-2 virus, save lives and protect the vulnerable.” To support countries to monitor implementation and evaluate progress, WHO subsequently developed the Global SPRP Monitoring and Evaluation Framework (27). WHO's early efforts at the country level were focused on policy dialogue to rapidly support countries to contextualize the global guidance and develop national country preparedness and response plans (CPRPs) (27).

The article "The World Health Organization's Frontline Support to Countries During the COVID-19 Pandemic in 2020" was published in 2022. Journal: Front Public Health.

By February 2020, 81% of WCOs had initiated support for developing CPRPs (10), with the proportion of countries with CPRPs increasing from 46% of all Member States in March 2020 to 83% in June 2020 (5) (Table 1). By the end of 2020, 91% of WHO Member States had CPRPs, and 119 were shared on the WHO Partners' Platform (5), a mechanism launched in March 2020 for real-time collaboration among countries, partners and donors (28) (Table 1).

During emergencies, WCOs support national authorities in data collection and analysis to enable strategic planning and decision-making based on quality and timely operational data. This was critical for SARS-CoV-2 as a new pathogen, and 71% of WCOs initiated support to national governments to develop a response monitoring framework before the first case of COVID-19 was reported in the country, and by March 2020, 77% of WCOs had provided support to develop and disseminate regular country situation reports and bulletins to partners and the public (10) (Table 1). In July 2020, WHO published guidance for countries in conducting Intra-Action Reviews (IARs) of national and subnational COVID-19 responses (30), with almost one quarter (36) of countries with a WCO conducting an IAR in 2020 (31).

Countries need robust health systems to effectively manage emergencies, and a core function of WCOs is to provide ongoing strategic support to Ministries of Health to maximize health system performance in terms of health results, equity and financial sustainability. Maintaining essential health services became a critical issue during the COVID-19 pandemic, with increased demand to care for people with COVID-19 and redeployment of the health workforce to COVID-19. By August 2020, almost all countries reported disruptions to essential health services such as mental health, reproductive and maternal health, routine childhood immunizations and nutrition services (32). To address these gaps, in May 2020, WHO included the maintenance of essential health services as a “pillar” in the operational planning guidance to support country preparedness and response (26) with WCOs providing strategic support to help countries implement the guidance. By April 2021, 87% of countries had developed a package of essential health services to be maintained during the pandemic, 82% of countries had designated a focal point, and 62% had allocated additional funding for the maintenance of essential health services (32) (Table 1).

The article "The World Health Organization's Frontline Support to Countries During the COVID-19 Pandemic in 2020" was published in 2022. Journal: Front Public Health.

WHO's policy dialogue and strategic health systems support to Nepal was critical in the early months of the pandemic as half a million Nepalese migrant workers returned home. WHO assisted with response efforts at the local level, by embedding staff and consultants in government units to provide rapid response to requests for support. This included analysis and interpretation of epidemiological and logistics data, with daily and weekly updates provided to government and stakeholders to support decision-making. Hospitals, laboratories, points of entries and local health units were assisted with implementing a digital system for case investigations, contact follow-up and transmission analyses. To address the decline in using essential health services including antenatal care, hospital deliveries and childhood vaccination, WHO focussed efforts on improving facility-based infection prevention and control measures and risk communication to improve safety and counter widespread misinformation among the community. With government and partners, WHO issued interim guidance to ensure the continuity of essential health services, supported the introduction of innovative health service delivery methods such as telemedicine, and provided technical guidance for establishing a COVID-19 call center (13).

## Technical Assistance and Service Delivery

One of WHO's core functions is to provide technical assistance to governments and partners on health topics and to build more robust technical capacities at country level (8). In 2020, WCOs prioritized technical assistance to build country capacity and support operationalization of CPRPs using the latest global guidance (10). WCOs drew on more than 500 guidance documents and scientific briefings developed by WHO on a range of topics including diagnostics, surveillance and clinical management that were incorporated into country level responses (5).

The article "The World Health Organization's Frontline Support to Countries During the COVID-19 Pandemic in 2020" was published in 2022. Journal: Front Public Health.

The provision of technical assistance to countries was hampered by public health, social and travel measures implemented to prevent COVID-19 transmission and therefore, WHO adapted its response model. Rather than send large-scale international deployments to countries as per the guidance for grade two and three emergencies (6), WHO mobilized and expanded its existing human resources on the ground. Across all WCOs, 60% of existing international staff were repurposed with more than 1,200 additional personnel rapidly recruited at the national level (10). Using this workforce, 84% of WCOs provided technical assistance to national governments and partners on priority interventions related to risk communication, community engagement and disease control measures before the first COVID-19 case was reported in the country (10) (Table 1). In addition, WHO utilized its existing interactive, online OpenWHO platform to further disseminate large-scale training to support operationalization of CPRPs, including on clinical management, infection prevention and control, laboratory and surveillance (33). By the end of 2020, there were more than 4.7 million enrollments and 2.5 million completed certificates issued by OpenWHO from the 22 courses on COVID-19 topics in 42 different languages (5).

WCOs used additional support mechanisms to meet the unprecedented demand for technical assistance in 2020. Nearly all countries with a WCO (93%) received in-person or virtual technical assistance from WHO experts based in regional or sub-regional offices, and 74% from experts at WHO headquarters (10). In addition, WHO leveraged its partnership networks, such as the Global Outbreak and Response Network (GOARN) (12) and Emergency Medical Teams (EMTs), the WHO-classified teams of health-care professionals. There were 191 deployments, which provided immediate assistance, training and support to countries in 2020 (5).

WHO, as the lead agency of the health cluster in humanitarian emergencies under the Inter-Agency Standing Committee, also has obligations to act as a “provider of last resort” of in-country services during emergencies (8). Originally, this mandate was expected to be required infrequently in a small subset of countries for a time limited period (8), however by February 2020, 83% of WCOs had initiated support for procurement and logistics due to the unprecedented challenges to the global supply chain caused by a rapidly spreading new SARS-CoV-2 virus (10) (Table 1). In April 2020, to accelerate development, production, and equitable access to COVID-19 medical countermeasures, WHO joined forces with governments, scientists, businesses, civil society, philanthropists and 8 other leading global health agencies to create the Access to COVID-19 Tools (ACT) Accelerator (34) and by September 2020, significant progress had been made in the development of effective new COVID-19 tests, treatments, and vaccines (35). At the country level, the minimum requirements for delivery of these COVID-19 tools was mapped in four of six WHO regions and 105 countries surveyed to identify potential bottlenecks and capacity gaps to inform planning and deployment (35). In 2020, WHO procured and supplied critical COVID-19 health commodities for 167 (86%) of its Member States (29), which included 16 thousand oxygen concentrators, 40 thousand oxygen monitors (5) as well as 200 million masks and millions more personal protective equipment (36) and by February 24, 2021, COVAX, the vaccines pillar of the ACT Accelerator commenced deployment of COVID-19 vaccines to participating economies (37).

The article "The World Health Organization's Frontline Support to Countries During the COVID-19 Pandemic in 2020" was published in 2022. Journal: Front Public Health.

WHO's provision of technical assistance and support for service delivery is well illustrated in the scaling-up of countries' laboratory capacities to test for SARS-CoV-2 and report cases to national surveillance systems. After January 13, 2020 when WHO published the first of several diagnostic molecular approaches for reverse transcription polymerase chain reaction (RT-PCR) assay to diagnose COVID-19 (38–43), countries rapidly developed testing capacities (5). WCOs provided technical assistance and training to laboratory technicians to implement the protocol and also supported procurement and shipping of 71 million diagnostic tests for 161 countries in 2020 through the COVID-19 Supply Chain System (5, 44). By March 2020, 85% of countries had access to laboratory testing (either in country or through an arrangement with a neighboring country) with all countries able to test for SARS-CoV-2 by the end of 2020 (5) (Table 1).

In February 2020, the WCO in Nigeria worked with national authorities and partners including the African Centers for Disease Control and Prevention to establish testing capacity for SARS-CoV-2 at the National Reference Laboratory (45). By the time the first case was confirmed on the February 27, 2020, five other laboratories in four states were conducting PCR testing for COVID-19 and by April 30, 2020, this had increased to 17 laboratories (45) with WHO support. The WCO supported the rollout of the national testing strategy for Nigeria, by providing technical assistance and training, not only to laboratory workers but also to health care workers across all 36 state governments, and supported service delivery by providing much needed reagents and consumables and transportation of samples (45, 46).

The article "The World Health Organization's Frontline Support to Countries During the COVID-19 Pandemic in 2020" was published in 2022. Journal: Front Public Health.

## Who's Strategy Delivered, But an Even Stronger Who is Needed in Countries for Future Emergencies

This article describes how WHO delivered the GPW13 through its country presence during the first year of the COVID-19 pandemic. WHO supported national authorities and partners through leadership, policy dialogue, strategic support, technical assistance, and service delivery at the country level. Despite these achievements, WHO identified several key challenges faced at the country level (10). Internal challenges included a lack of flexible funding and insufficient technical capacities available on the ground for WHO to meet specific needs. Country-related challenges included limited preparedness for response and in some cases, delayed or restricted access to information and data. Insufficient collaboration with partners and overlapping efforts, plus operational challenges due to response measures, such as widespread lockdowns and a global supply chain disruption, were also documented (10).

In July 2021, a representative Member States Working Group on Strengthening WHO Preparedness and Response to Health Emergencies (WGPR) was established (17) to consider the feasibility and impact of implementation of the collective 131 recommendations from three independent reviews (14–16), as per World Health Assembly resolution (WHA74.7, 2021) (47). Agreeing that “the status quo is unacceptable for everyone” the WGPR has generated broad consensus on the importance of strengthening the role of WHO in health emergencies and a shared commitment to strengthen global, regional, and national preparedness and response (17). A total of 44 recommendations are under consideration to strengthen WHO's core functions in the following areas: (1) providing adequate resources for WCOs to respond to requests from national governments; (2) supporting Member States to develop and operationalize disease-specific strategies and plans for pandemic preparedness and response that include measurable targets and benchmarks and ensure full implementation of the core capacities required by the International Health Regulations (2005); (3) coordinating the WHO Secretariat's technical, normative, and managerial work across all three levels of the Organization; (4) supporting access to timely, accurate, and easy-to-understand advice and information on public health events; (5) promoting, advocating and/or supporting Member States to implement whole-of-government and whole-of-society approaches to strengthen pandemic preparedness and response, and; (6) working with partners to develop and implement mechanisms that promote fair and equitable access to pandemic supplies and countermeasures (17). These improvements will address the challenges of the first year of the COVID-19 response and better equip WHO to provide more effective support to countries' emergency preparedness and response and the development of stronger and more resilient health systems.

The article "The World Health Organization's Frontline Support to Countries During the COVID-19 Pandemic in 2020" was published in 2022. Journal: Front Public Health.

The WGPR will submit a report with proposed actions for consideration by the seventy-fifth World Health Assembly in May 2022 (17). As the COVID-19 pandemic continues to have global impact and severely impede progress toward the sustainable development goals, and the real threat of new and potentially more infectious strains of SARS-CoV-2 and other health emergencies loom, there is no time to lose in reinforcing WHO's country offices as the frontline of support to its Member States.

## Data Availability Statement

The original contributions presented in the study are included in the article/supplementary material, further inquiries can be directed to the corresponding author/s.

## Author Contributions

AC, KW, CH, PG, and SA: conceptualization. KW, CH, AC, and OO: data collection and interpretation. CH, AC, MM, and KW: drafting the manuscript. KW, CH, AC, OO, MM, SA, and PG review and revising manuscript. All authors contributed to the article and approved the submitted version.

## Conflict of Interest

The authors declare that the research was conducted in the absence of any commercial or financial relationships that could be construed as a potential conflict of interest.

## Publisher's Note

All claims expressed in this article are solely those of the authors and do not necessarily represent those of their affiliated organizations, or those of the publisher, the editors and the reviewers. Any product that may be evaluated in this article, or claim that may be made by its manufacturer, is not guaranteed or endorsed by the publisher.
